# Heme Oxygenase-2 Localizes to Mitochondria and Regulates Hypoxic Responses in Hepatocytes

This article has been retracted.

**DOI:** 10.1155/2018/2021645

**Published:** 2018-04-12

**Authors:** Paul K. Waltz, Benjamin Kautza, Jason Luciano, Mitch Dyer, Donna Beer Stolz, Patricia Loughran, Matthew D. Neal, Jason L. Sperry, Matthew R. Rosengart, Brian S. Zuckerbraun

**Affiliations:** ^1^Department of Surgery, University of Pittsburgh, Pittsburgh, PA, USA; ^2^Department of Cell Biology, University of Pittsburgh, Pittsburgh, PA, USA; ^3^Center for Biologic Imaging, University of Pittsburgh, Pittsburgh, PA, USA; ^4^Department of Critical Care Medicine, University of Pittsburgh, Pittsburgh, PA, USA; ^5^VA Pittsburgh Healthcare System, Pittsburgh, PA, USA

## Abstract

Hypoxia occurs as a part of multiple disease states, including hemorrhagic shock. Adaptive responses occur within the cell to limit the consequences of hypoxia. This includes changes in mitochondrial respiration, stress-induced cell signaling, and gene expression that is regulated by hypoxia inducible factor-1*α* (HIF-1*α*). Heme oxygenase-2 (HO-2) has been shown to be involved in oxygen sensing in several cell types. The purpose of these experiments was to test the hypothesis that HO-2 is a critical regulator of mitochondrial oxygen consumption and reactive oxygen species (ROS) production to influence hypoxia-adaptive responses such as HIF-1*α* protein levels and JNK signaling. *Methods and Results*. *In vitro* studies were performed in primary mouse hepatocytes. HO-2, but not HO-1, was expressed in mitochondria at baseline. Decreased oxygen consumption and increased mitochondrial ROS production in response to hypoxia were dependent upon HO-2 expression. HO-2 expression regulated HIF-1*α* and JNK signaling in a mitochondrial ROS-dependent manner. Furthermore, knockdown of HO-2 led to increased organ damage, systemic inflammation, tissue hypoxia, and shock in a murine model of hemorrhage and resuscitation. *Conclusion*. HO-2 signaling plays a role in hypoxic signaling and hemorrhagic shock. This pathway may be able to be harnessed for therapeutic effects.

## 1. Introduction

Tissue and cellular hypoxia are components of many disease processes, including shock states and ischemia/reperfusion insults. Molecular oxygen can be considered an essential nutrient and acts as a substrate in many biological processes, not the least of which is the terminal electron acceptor in the electron transport chain to produce ATP [1, 2]. Perturbations in oxygen levels can potentially disrupt oxygen-dependent reactions; however, many adaptive responses occur to regulate bioenergetic and oxygen demands in response to alterations in the availability of oxygen. In the setting of hypoxia, critical mammalian cellular processes are temporarily limited to reduce energy consumption. Furthermore, cells adapt by initiating survival signaling responses including hypoxia-inducible factor-based signaling, autophagy, and the unfolded protein response [3–7].

The pathophysiology of multiple disease processes, including hemorrhagic shock or ischemia/reperfusion, is driven by tissue hypoxia. Understanding the signaling mechanisms that occur as a result of hypoxia during these disease processes is essential for novel therapeutic development.

Heme oxygenase (HO) enzymes, which are the rate-limiting enzymes in the breakdown of heme to free iron, biliverdin, and carbon monoxide (CO), are critical to the maintenance of cellular homeostasis [8, 9]. HO enzymes have been implicated in the sensing of oxygen levels and the regulation of oxygen consumption. HO-1, presumably through the production of CO, can limit cellular respiration and cytochrome C oxidase activity [10–12]. Moreover, HO-2, which is constitutively expressed in many cell types, has been shown to be a critical oxygen sensor in glomus cells of the carotid body that influence the respiratory rate via interaction with the large conductance potassium channel [13–15].

Mitochondria act as rheostats within a cell to orchestrate cellular responses to various stimuli, including hypoxia [16]. These changes regulate mitochondrial dynamics and structure, as well as mitochondrial signaling such as reactive oxygen species (ROS) generation. Oxygen levels influence such responses, but relative levels of other gases such as CO and nitric oxide (NO) that compete for oxygen-binding sites on enzymes such as cytochrome C oxidase may also influence oxygen signaling [1]. The purpose of these investigations was to test the hypothesis that HO-2 is protective against the development of shock and organ injury in hemorrhagic shock and to test the hypothesis that HO-2 serves as a critical regulator of hypoxic responses in hepatocytes via modulation of mitochondrial signaling.

## 2. Methods

### 2.1. Cell Culture

Primary mouse hepatocytes were harvested from C57BL/6 mice. They were cultured in William E media supplemented with penicillin (100 U/ml), streptomycin (100 *μ*g/mL), insulin (0.16 mL), HEPES buffer (7.5 mL) (Gibco), and 5% calf serum (Gibco, Gaithersburg, MD) on either gel-coated plates for protein extraction or on cover slips for immunohistochemistry. Cells were utilized on day 2 of harvest. Heme-oxygenase was inhibited with tin protoporphyrin (SnPP) (50 *μ*M) (Frontier Scientific, Logan, UT), a known, nonspecific inhibitor of HO-, or HO-1-, or HO-2-specific siRNA (50 *μ*M) (Invitrogen, Waltham, MA).

### 2.2. Hemorrhagic Shock Model

The University of Pittsburgh Institutional Animal Care and Use Committee approved animal protocols. The experiments were performed in adherence to the National Institutes of Health Guidelines on the Use of Laboratory Animals. Hemorrhagic shock was performed as described previously [17–21]. Briefly, C57BL/6 mice weighing 23 to 27 g were anesthetized with pentobarbital (70 mg/kg i.p). The right and left femoral arteries were cannulated. The left arterial catheter was connected to a monitor to follow the mean arterial pressure (MAP) and heart rate. Blood was withdrawn for more than 10 min via the right femoral artery to achieve a MAP of 25 mmHG for a total of 120 minutes. Sham animals were cannulated but were not subjected to hemorrhage. At the end of the shock period, mice were resuscitated with Ringer's lactate solution using a total of two times the volume of maximum shed blood. Sham mice were subject to the same surgical procedure but did not undergo hemorrhage and did undergo resuscitation. Four hours after the onset of resuscitation, the mice were killed and serum and organs were collected.

Experiments assessing time until cardiovascular collapse and arterial pH were performed similar to that described above; however, blood was withdrawn to reach a MAP of 20 mmHg. The duration of time that mice were able to maintain a MAP of 20 mmHg without return of volume was assessed, at which time the mice were sacrificed and arterial blood and organs were collected.

HO was inhibited *in vivo* with the use of *in vivo* HO-1- or HO-2-specific small interfering RNA [siRNA; 50 *μ*M/kg] (Invitrogen, Waltham, MA). This was administered via hydrodynamic tail vein injection where the siRNA was made to the correct concentration in 2 cc of lactated ringers and given 48 hours prior to hemorrhagic shock as described previously [22]. The rapid injection of this large volume creates significant pressure to help promote siRNA uptake. Scramble siRNA (50 *μ*M/kg) was utilized as a control again via hydrodynamic tail vein injection.

### 2.3. Serum Cytokine and Alanine Aminotransferase Measurement

ELISA kits (Abcam, Cambridge, MA) were used according to the manufacturer's instructions to measure the levels of cytokines interleukin 6 (IL-6) and tumor necrosis factor-*α* (TNF-*α*). Serum alanine aminotransferase (ALT) was measured with Heska DRI-Chem 4000 (Heska, Tokyo, Japan).

### 2.4. Western Blotting

Western blots were performed on liver tissue or hepatocytes. Proteins were separated by sodium dodecyl sulfate polyacrylamide gel electrophoresis and transferred onto a nitrocellulose membrane. The membrane was blocked for 1 hour in TBS-Tween 20 with 5% milk, followed by immunostaining with dilutions of primary antibodies [mouse anti-HIF-1a (Novus, Littleton, CO), rabbit anti-HO-2 (Abcam), rabbit anti-HO-1 (Affinity Biosciences, Cincinnati, OH), mouse anti-COX IV (Abcam), mouse anti-beta actin (Abcam), and rabbit anti-total or mouse anti-phospho JNK (Cell Signaling Technology, Danvers, MA)] in 1% milk in phosphate-buffered saline- (PBS-) Tween from 1 hour to overnight at 4°C. Secondary antibodies conjugated with horseradish peroxidase and washed for 1 hour in TBST before being developed with the SuperSignal West Pico chemiluminesence kit (Thermo Fisher Scientific, Waltham, MA). Beta actin was used as a loading control for all whole cell experiments.

### 2.5. Immunocytochemistry/Immunohistochemistry

Hepatocytes were rinsed twice with cold PBS, then fixed on cover-slips with 2% paraformaldehyde for 15 minutes. Slides were subsequently stained for monoclonal mouse anti-HIF-1*α* (Novus) or polyclonal rabbit anti-HO-2 (Abcam). Secondary antibodies for goat anti-rabbit or anti-mouse conjugated to Cy5 were utilized. For experiments using MitoTracker Green (Thermo Fisher) or hypoxyprobe [mouse IgG1 monoclonal antibody conjugated to fluorescein (HP-FITC-MAb) and pimonidazole; Hypoxyprobe, Burlington, MA], these were added to the cells 30 minutes prior to fixation with paraformaldehyde. Images were taken with a Zeiss 510 inverted confocal microscope.

For immunohistochemistry and measurement of *in vivo* relative oxygen levels, EF5 (Hypoxia Imaging Group, University of Pennsylvania) delivery and staining were performed as previously described [23]. EF5 was injected intraperitoneally 15 min before the initiation of shock. Liver tissue from mice was removed after perfusion with cold PBS and 2% paraformaldehyde. Tissue was then placed in paraformaldehyde for one hour then switched to 30% sucrose solution for 12 hours. The tissue was then slowly frozen in 2-methylbutane. Seven-micron sections were obtained. Sections were stained using antibodies against EF5 protein-binding adducts.

### 2.6. Electron Microscopy

Hepatocytes were fixed and embedded by inverting Polybed 812-filled Better Equipment for Electron Microscopy (BEEM) capsules on top of the cells. Blocks were cured overnight at 37°C and then cured for two days at 65°C. Monolayers were pulled off the plastic and re-embedded for cross-sectioning. Ultrathin cross sections (60 nm) of the cells were obtained on a Reichert Ultracut E microtome. Sections were washed three times with PBS and three times with PBS containing 0.5% bovine serum albumin and 0.15% glycine (PBAG), followed by a 30 min incubation with 5% normal goat serum in PBAG. Sections were labeled with polyclonal anti-rabbit HO-2 (Abcam; 1 : 50) in PBG for 1 h. Sections were washed four times in PBAG and were labeled with goat anti-rabbit (10 nm) gold-conjugated secondary antibodies (Amersham, Piscataway, NJ), each at a dilution of 1 : 25 for 1 h. Sections were washed three times in PBAG and three times in PBS and were then fixed in 2.5% glutaraldehyde in PBS for 5 min, washed two times in PBS, then washed six times in sterile water. Sections were poststained in 2% neutral uranyl acetate for 7 min, washed three times in sterile water, stained for 2 min in 4% uranyl acetate, and then embedded in 1.25% methyl cellulose. Labeling was observed on an electron microscope (JEM 1210; JEOL, Peabody, MA) at 80 kV.

### 2.7. Statistical Analysis

Results are expressed as mean ± standard error of the mean (SEM). SigmaPlot (Systat Software, Inc., Point Richmond, CA) was used for statistical analysis using either Student's *t*-test for pairwise comparisons or one-way analysis of variance for significance and Tukey's post hoc test. Significance was established at *P* < 0.05. All *in vitro* experiments were performed in triplicate and repeated three times. All *in vivo* experiments contained 6–8 mice per group as specified.

## 3. Results

### 3.1. HO-2 but Not HO-1 Is Expressed in Hepatic Mitochondria at Baseline

HO-2 localizes to mitochondria in unstimulated hepatocytes as determined by immunohistochemistry and electron microscopy (Figures 1(a) and 1(b)). Additionally, Western blotting of mitochondrial fractions of hepatocytes in culture or mouse liver reveals that HO-2 protein, but not HO-1 protein, is present within the mitochondria in unstimulated conditions (Figures 1(c) and 1(d)) Mitochondrial cytochrome C oxidase subunit 4 (COX IV) is used as a mitochondrial loading control.

### 3.2. Knockdown of HO-2 Increases Hypoxia-Induced Oxygen Consumption and Decreases Cellular Oxygen Levels

The influence of heme oxygenase enzymes on oxygen consumption is presumably secondary to CO production and decreased activity of cytochrome C oxidase. HO-1 overexpression or CO exposure can limit oxygen consumption and decrease cellular hypoxia in hepatocytes [23]. However, given that HO-2 (and not HO-1) is expressed at baseline and localizes to mitochondria, the constitutively expressed HO-2 may be more relevant than HO-1 for physiologic perturbations in oxygen levels or initial hypoxic stress. The influence of 1% oxygen on heme oxygenase enzymatic activity was measured to determine if these enzymes are active at low oxygen concentrations and can contribute to cell signaling under these conditions. HO activity was maintained at 1% oxygen levels and was decreased by SnPP or HO-2 siRNA in both normoxic and hypoxic conditions (Figure 2(a)). Hepatocyte oxygen consumption was decreased in cells exposed to 1% oxygen (Figure 2(b); 68.5 ± 11.9% in vehicle controls and 60.8 ± 14.9% in siRNA controls compared to vehicle controls in normoxia; ^∗^*P* < 0.05). Treatment with SnPP, to nonspecifically inhibit HO activity, prevented this decrease in the rate of oxygen consumption (96.9 ± 10.4% compared to vehicle controls in normoxia; ^#^*P* < 0.05 compared to vehicle controls in hypoxia). Similarly, knockdown of HO-2, but not HO-1, prevented this change in oxygen consumption with acute exposure to 1% oxygen (Figure 2(b); 89.7 ± 22.3% in HO-2 siRNA in hypoxia and 58.8 ± 10.4% in HO-1 siRNA in hypoxia compared to vehicle controls in normoxia). Intracellular oxygen levels were determined under 21% or 1% oxygen with control or HO-2 siRNA using hypoxyprobe staining. Relative intracellular hypoxia was exacerbated with HO-2 siRNA treatment as demonstrated by increased hypoxyprobe staining (Figure 2(c)). Additionally, hypoxia is known to increase mitochondrial production of ROS thought to be secondary to the decreased availability of oxygen as a terminal electron acceptor in the electron transport chain. Hypoxia increased relative MitoSOX fluorescence at 20 minutes by 149 ± 7% and increased to 223 ± 10% at 60 minutes (*P* < 0.05 compared to normoxic controls). Hypoxia-induced production of ROS was inhibited by HO-2 siRNA (Figure 2(d); maximal relative fluorescence at 60 minutes increased to 137 ± 5% of baseline). Furthermore, hypoxia-induced ROS generation was similar in hepatocytes harvested from wild-type mice and from *gp91phox^−/−^* mice (data not shown), further suggesting that these changes in intracellular ROS levels were mitochondrial in origin and not contributed by NADPH oxidase. Taken together, these data indicate that HO-2 is a critical regulator of oxidative phosphorylation and mitochondrial function.

### 3.3. HO-2 Influences Hypoxia-Inducible Factor 1-Alpha (HIF-1*α*) Stabilization

Given the apparent influence of HO-2 on the regulation of oxygen consumption in hepatocytes, the influence on HIF-1*α* stabilization was determined. Western blot analysis of hepatocytes pretreated with SnPP or with HO-2 siRNA demonstrated decreased hypoxia-induced HIF-1*α* stabilization (Figures 3(a)–3(c)). Hypoxia increased HIF-1*α* protein levels, and nuclear localization was also demonstrated by immunocytochemistry for HIF-1*α* (Figure 3(d)). Increased activation of a HIF-1*α* luciferase reporter assay by 4.36 ± 0.68 (*P* < 0.05) over normoxia also confirmed these findings (Figure 3(f)). HO-2 siRNA treatment limited these hypoxia-induced effects on HIF-1*α*. HO-2 siRNA limited HIF-1*α* luciferase reporter activation under hypoxic conditions, leading to only a 1.64 ± 0.61-fold increase over baseline (*P* < 0.05 compared to hypoxic controls). Mitochondrial ROS scavenging by MitoTEMPO limited hypoxia-induced HIF-1*α* stabilization as determined by immunocytochemistry and luciferase reporter assay (Figures 3(e) and 3(f)). MitoTEMPO limited hypoxia-induced increases in HIF-1*α* luciferase reporter activation, resulting in a 1.92 ± 0.73-fold increase over baseline (*P* < 0.05 compared to hypoxic controls).

### 3.4. HO-2 Modulates Downstream (JNK) Signaling

Based upon the ability of HO-2 to modulate intracellular oxygen consumption and mitochondrial ROS generation, we next sought to investigate whether HO-2 might play a role in modulating the stress signaling JNK pathway. As shown previously [24], these data confirm that hypoxia leads to increased JNK phosphorylation in hepatocytes (Figure 4(a)). Inhibition of HO activity or knockdown of HO-2 blunted the increase in JNK phosphorylation under hypoxic conditions (Figures 4(b) and 4(c)). The influence on hypoxia-induced ROS production on JNK activation was determined by measuring JNK phosphorylation under hypoxia with the addition of the mitochondrial targeted ROS scavenger, MitoTEMPO (Figure 4(d)). Taken together, these results suggest that HO-2 influences oxidative phosphorylation to increase mitochondrial ROS in hypoxia, which then acts as a second messenger to activate downstream signaling, including JNK.

### 3.5. Inhibition of HO-2 Is Associated with Exacerbation of Tissue Injury and Worsened Clinical Outcome in a Murine Model of Hemorrhagic Shock/Resuscitation

Hemorrhagic shock and resuscitation result in relative tissue ischemia followed by reperfusion and result in organ injury and systemic inflammation. In the setting of hemorrhagic shock, HO-2 knockdown was associated with an exacerbation of systemic inflammation as well as worsened hepatic injury as determined by serum ALT, IL-6, and TNF-*α* levels (Figures 5(a)–5(c)). Mice pretreated with HO-2 siRNA demonstrated worse hepatic hypoxia by EF5 staining compared to control siRNA-treated mice (Figure 5(d)). Furthermore, mice with HO-2 siRNA had worse parameters of shock, as determined by a shortened time to compensation endpoint (the time point in the hypotensive period when they were no longer able to maintain a MAP of 20 mmHg without the return of fluid) and an increased degree of arterial acidosis at 20 minutes into the hypotensive period (Figures 5(e) and 5(f)). Control mice undergoing shock reached compensation endpoint at 42.8 ± 3.1 minutes. Mice receiving SnPP or HO-2 siRNA reached the compensation endpoint at earlier time points (29.1 ± 4.2 and 30.9 ± 3.0 minutes, respectively; *P* < 0.05 compared to control shock mice). Using arterial pH as a clinical parameter of shock demonstrates that hemorrhage results in a lower pH compared to control mice (7.32 ± 0.05 versus 7.18 ± 0.08 in shock control siRNA; *P* < 0.05). HO-2 siRNA-treated mice demonstrated exacerbated academia (7.03 ± 0.06; *P* < 0.05 versus shock control siRNA mice).

## 4. Discussion

There is a significant body of literature on heme oxygenases and the protective roles that these enzymes play within the cell [9, 25]. The vast majority of this research, particularly in stress states, has primarily focused on the inducible heme oxygenase homolog, HO-1, and much less on the constitutively expressed HO-2. These data demonstrate that HO-2 is present in the mitochondria of hepatocytes and influences oxygen consumption. Additionally, since HO-2 is expressed at baseline, this enzyme may regulate early responses to physiologic and pathophysiologic perturbations in oxygen levels.

Similar to previous studies that examined a protective role of HO-2 in the brain, we have shown that knockdown of HO-2 is associated with an exacerbated inflammatory cytokine profile and worsened hepatic tissue injury in a murine model of hemorrhagic shock and resuscitation. These findings are in line with work done by DorÃ et al. who noted an increased severity of ischemia on neuronal injury and brain swelling in *hmox2^−/−^*mice in comparison to *hmox1^−/−^* mice [26]. These authors hypothesized that this may be secondary to influences on circulatory compensation. Although the protective effects of endogenous HO-2 may be secondary in part to influences on the microcirculation, this was not examined in our study. The increase in TNF-*α* and IL-6 that we have shown following hemorrhagic shock with HO-2 knockdown is additionally consistent with findings of an exacerbated inflammatory cytokine profile expression from aortic endothelial cells seen in *hmox2^−/−^*mice [27].

These data suggest a role for HO-2 as an oxygen sensor within the cell. This is supported by the findings that under acute hypoxic conditions, nonspecific inhibition of HO activity or HO-2 knockdown (but not HO-1 knockdown) prevents the hypoxia-induced slowing of oxygen consumption, limits the production of mitochondrial ROS, and prevents increases in HIF-1*α* levels. The exact mechanism for HO-2 oxygen sensing is not completely understood; however, the influence on mitochondrial oxygen consumption to regulate overall intracellular oxygen availability has the potential to influence other cellular oxygen-dependent processes. Another hypothesis involves heme-binding motifs outside of the catalytic site on HO-2 that function as molecular rheostats [28–30]. The heme-binding motifs possess cysteine residues that are redox sensitive and can form a disulfide bridge releasing free heme and/or increasing the catalytic activity of HO-2. This has been suggested to influence potassium channel signaling. Furthermore, it has been suggested that HO-2 functions in glomus cells as an oxygen sensor based upon oxygen-dependent CO production to regulate the BK potassium channel [15]. As a contradiction to these previous studies, the current data does not show that HO activity is sensitive to the acute changes in oxygen levels in hepatocytes at 1% oxygen *in vitro*. It is possible that with changes in oxygen tension, the heme recognition motifs serve as a redox switch to release heme directly to the catalytic site in HO-2 or to other locations in the cell to influence biological processes.

HO-2 has also been shown to play a role in the regulation of extracellular superoxide dismutase and in turn the extracellular redox state [31]. These data in the current study have shown that HO-2 modulates intracellular and specifically mitochondrial ROS generation induced by hypoxia. Additionally, these data suggest that hypoxia-induced intracellular ROS are not NADPH oxidase mediated based upon the unaltered intracellular production of ROS in *gp91phox^−/−^* hepatocytes.

HO-1 and ROS have previously been shown to affect mitogen-activated protein kinase (MAPK) signaling as well as the transcription factor nuclear factor-kappa B (NF-*κ*B) signaling [32, 33]. Not much is known regarding HO-2 and its ability to modulate adaptive signaling pathways following hypoxia. These data would suggest that the phosphorylation of JNK in hypoxia is via an HO-2-mitochondrial ROS signaling pathway.

This study adds to the growing body of literature showing the protective role of HO-2. These data show that HO-2 modulated the inflammatory cytokine profile and severity of hepatic injury following hemorrhagic shock. Given its constitutive presence within hepatocytes and specifically its presence within the mitochondria at basal conditions, HO-2 is able to play a critical oxygen-sensing role within the cell leading to alterations in cellular ROS production and downstream adaptive signaling. Manipulation of HO-2 signaling or perhaps the therapeutic delivery of CO as a biologically active product of HO signaling may prove to be a useful strategy to treat hemorrhagic shock or other conditions involving tissue hypoxia in the future.

## Figures and Tables

**Figure 1:** HO-2 is present within hepatocyte mitochondria under unstressed conditions. (a, b) Microscopy reveals localization of HO-2 within the mitochondria. Immunocytochemistry (a) demonstrates mitochondria (green; MitoTracker) and HO-2 (red) with areas of yellow representing colocalization. Immunoelectron microscopy demonstrates gold particle-labeled localization of HO-2 within hepatocyte mitochondria under normal cell culture conditions (b). (c, d) Western blot of mitochondrial fractions of untreated primary hepatocytes (c) and mouse liver (d) demonstrates HO-2 but not HO-1 expression protein levels under basal cell culture or without treatment. Mitochondrial cytochrome C oxidase subunit 4 (COX IV) is used as a mitochondrial loading control.

**Figure 2:** HO-2 regulates oxidative phosphorylation in hypoxia. (a) Hepatocyte heme oxygenase activity is not influenced significantly by hypoxia and is diminished by tin protoporphyrin (SnPP) or HO-2 siRNA. ^∗^*P* < 0.05 compared to control siRNA in 21% O_2_. (b) Oxygen consumption is decreased in hepatocytes under hypoxic conditions, and this is reversed by nonspecific pharmacological inhibition of HO activity or knockdown of HO-2, but not HO-1. ^∗^*P* < 0.05 compared to vehicle controls in 21% O_2_; ^#^*P* < 0.05 compared to vehicle controls in 1% O_2_. (c) Hypoxyprobe staining increases with decreased availability of intracellular oxygen. Hypoxyprobe staining increases under hypoxic conditions and increases further with knockdown of HO-2 (suggesting increased cellular hypoxia). (d) Mitochondrial ROS increases under hypoxia in hepatocytes as determined by relative MitoSOX fluorescence. This is reversed by knockdown of HO-2.

**Figure 3:** Hypoxia-induced HIF-1*α* stabilization is dependent in part on HO-2 and mitochondrial ROS. (a) HIF-1*α* protein levels are increased in hepatocytes following 90 minutes of hypoxia. (b) Inhibition of HO activity with tin protoporphyrin (SnPP) limits hypoxia-induced increases in HIF-1*α* protein levels. (c–f) HO-2 siRNA decreases hypoxia induces HIF immunocytochemistry (d) and 1-*α* levels as determined by Western blotting (c) and luciferase-reporter assay (f). Furthermore, inhibition of mitochondrial ROS production by MitoTEMPO also decreases HIF-1*α* as determined by immunocytochemistry (e) and luciferase-reporter assay (f). ^∗^*P* < 0.05 compared to control siRNA 21% O_2_; ^#^*P* < 0.05 compared to control siRNA 1% O_2_.

**Figure 4:** Hypoxia-induced JNK phosphorylation is partially dependent on HO-2 and mitochondrial ROS production. (a) Phosphorylated JNK (p-JNK) is increased in hepatocytes following 90 minutes of hypoxia. (b) Inhibition of HO activity with tin protoporphyrin (SnPP) limits hypoxia-induced increases in phosphorylation of JNK. (c) HO-2 siRNA limits phosphorylation of JNK during a one-hour time course of hypoxia treatment. (d) Treatment with MitoTEMPO to limit mitochondrial ROS generation decreases hypoxia-induced JNK phosphorylation at a 60-minute time point.

**Figure 5:** Inhibition of HO-2 exacerbates injury and inflammation in a murine hemorrhagic shock model. (a, b) Knockdown of HO-2 exacerbates hemorrhagic shock-induced serum TNF-*α* (275 ± 56 control siRNA versus 387 ± 67 HO-2 siRNA) and IL-6 (621 ± 87 control siRNA versus 903 ± 91 HO-2 siRNA). Units are pg/mL; ^∗^*P* < 0.05 compared to sham mice and ^#^*P* < 0.05 compared to shock control siRNA mice. *N* = 6 mice per group. (c, d) Liver injury and hypoxia were worse in the setting of knockdown of HO-2. Serum ALT increased from 225 ± 59 to 573 ± 102 IU/mL; *n* = 6 mice per group (c). Hemorrhagic shock also resulted in increased tissue hypoxia as demonstrated by staining for the nitroimidazole EF5, which was also increased by HO-2 siRNA pretreatment (d). (e) Knockdown of HO-2 or nonspecific inhibition of HO activity is associated with earlier decompensation in severe hemorrhagic shock (MAP 20 mmHg). *N* = 6 mice per group. (f) Arterial pH 30 minutes into severe hemorrhagic shock is decreased compared to control mice (7.32 ± 0.05 versus 7.18 ± 0.08 in shock control siRNA; ^∗^*P* < 0.05). This clinical shock parameter is further decreased in HO-2 siRNA-treated mice (7.03 ± 0.06; ^#^*P* < 0.05 versus shock control siRNA mice). *N* = 8 mice per group.
